# Clinical Effect of the Treatment of Lumbar Intervertebral Disc Protrusion

This article has been retracted.

**DOI:** 10.1155/2022/6803124

**Published:** 2022-04-29

**Authors:** Yehui Zhou, Ming Yang

**Affiliations:** Wuhan No.4 Hospital, WuHan 430000, China

## Abstract

Compared with traditional acupuncture, it is urgently needed for more effective method for the disease to serve the clinical treatment. This paper combines acupuncture and massage to treat lumbar intervertebral disc protrusion, uses a controlled trial to study the clinical effects of acupuncture combined with massage for the treatment of lumbar intervertebral disc protrusion, combines mathematical statistics to test the data, and compares and analyzes the statistical object parameters. Through experimental research, it is known that in the treatment of lumbar intervertebral disc protrusion, in order to obtain a faster and better effect, traditional acupuncture treatment should be combined with massage therapy. On the basis of fully eliminating the pathological factors, the intervertebral disc is reset by mechanical treatment, which makes the patient more likely to heal. Therefore, it is a comprehensive treatment plan that is worth adopting.

## 1. Introduction

Lumbar intervertebral disc protrusion (LIDP) is caused by fissures in the lumbar intervertebral annulus degeneration or trauma. Under the action of external force, the nucleus pulposus and other intervertebral disc tissues bulge or protrude backward or rearward to stimulate and compress the spinal cord nerve roots. Furthermore, nerve root inflammation, nerve root dystrophy, and conduction damage are caused, and there are low back pain, sciatica, and even obvious nerve dysfunction.

The population prediction findings reveal that, as the number of persons involved in mental work and light industries in China increases, the incidence of this illness is growing year by year, owing to variables such as long-term sitting job and less physical activity. In both domestic and international medicine, there are several therapeutic options for lumbar intervertebral disc protrusion, which may be loosely split into two categories: surgical therapy and nonsurgical therapy [1]. According to statistics, active and suitable nonsurgical treatments, such as medicine, acupuncture, massage, lumbar traction, and physical therapy, may cure or ease 85 percent to 90 percent of patients with lumbar intervertebral disc protrusion. For lumbar intervertebral disc protrusion, acupuncture is a nonsurgical therapeutic option. There are several clinical studies and procedures available. It has a unique healing effect, is simple to operate, is cost-effective, is safe, is less uncomfortable, and has less adverse responses, among other qualities that have been extensively acknowledged [2]. There are different acupuncture points, heavy acupuncture and light moxibustion, and different operations. Therefore, how to select acupoints, optimize acupuncture prescriptions, give full play to the characteristics of acupuncture and moxibustion, and standardize technical operations to further improve the clinical efficacy of this disease is still worth studying [3].

The disease should be classified into the categories of “back pain,” “back and leg pain,” and “arthralgia” in traditional medicine. The occurrence of low back pain is most closely related to the bladder meridian and the governor channel. The foot and bladder meridian “has the ridge to the waist,” while the governor channel is “in the spine.” Therefore, the differentiation and treatment of low back pain cannot be separated from the bladder meridian and the governor channel. The occurrence of this disease is based on the inherent prerequisite of the inherent weakness of the congenital endowment and the external cause of feeling wind, cold, dampness, and heat. Internal injury and weakness, external pathogenic qi, and injury and stasis are the key pathological reasons in this condition, which produce muscle and vein constriction and loss of waist nutrition. Traditional Chinese medicine has a long history of treating low back pain and has a surprising therapeutic impact. The therapy approach offers unique benefits and is irreplaceable, and it is always being refined and enhanced. It mostly consists of oral Chinese medicine, external Chinese medicine therapy, acupuncture, and moxa. Moxibustion, massage, cupping, fire needles, tiny needle knives, and other techniques are used. Acupuncture and massage were used to treat lumbar intervertebral disc herniation in this research. We are searching for a more successful way for the ailment than conventional acupuncture, so we can better serve the clinical therapy.

## 2. Related Work

At present, there are many treatment methods for lumbar intervertebral disc herniation, which generally include conservative treatments such as acupuncture and massage, minimally invasive treatments such as chemical nucleolysis, and surgical treatments. Because conservative treatment has the advantages of low cost and high safety, most patients choose conservative treatment as the main treatment, using acupuncture, massage, traction, drugs, and other methods for treatment. As a common therapy in conservative treatment, acupuncture can increase the patient's pain threshold, improve local and surrounding blood circulation, quickly eliminate nerve root edema, and promote the absorption of local aseptic inflammation. Because of its definite curative effect, high safety factor, and low pain, it is accepted by the majority of patients.

Western medicine has not yet fully understood the etiology and pathogenesis of lumbar intervertebral disc herniation. The fibrous ring, which plays an important role in the pathogenesis of lumbar intervertebral disc herniation, also consists of a three-layer structure. The outer layer is collagen fibers, and the middle and inner layers are cartilage fibers. Among all the vertebral bodies of the spine, the lumbar spine has the highest weight-bearing strength. It is functionally determined that its vertebral bodies are the thickest among all vertebral bodies and are arranged in a flat top and bottom structure. The present etiology is mostly influenced by lumbar spine degenerative causes, mechanical tissue compression, and neuroinflammatory responses. Different treatments for managing lumbar disc herniation have been developed based on the aforementioned pathophysiology, which are primarily separated into surgical therapy and nonsurgical treatment. According to research, 80 percent of individuals with lumbar disc herniation may manage their symptoms and improve their function with nonsurgical therapy, either alone or in combination. Anti-inflammatory analgesics, neurotrophic medications, and steroid hormones are the mainstays of pharmacological treatment, with anti-inflammatory analgesics, neurotrophic drugs, and steroid hormones being the most common. Many therapies between medications and surgical treatments have been developed as a result of contemporary medicine's invention and progress, including ozone interventional therapy, radiofrequency ablation, and nerve block surgery.

A great number of research have indicated that acupuncture for lumbar intervertebral disc protrusion is useful in reducing pain. The strategy of integrating local lesions with distant acupoint selection along the meridian and dialectical matching of acupoints has a greater cure rate in clinical acupoint selection. Selecting neighboring acupoints may assist remove or decrease nerve root inflammation and edema by improving local blood circulation, promoting tissue metabolism, and eliminating or reducing nerve root inflammation and edema. Remote access and point selection based on syndrome distinction may also help with analgesia and systemic symptoms. A total of 160 patients with LIDP were randomly assigned to an acupuncture group with 80 cases and a medication group with 80 cases, according to the literature [4]. Acupuncture along the meridian was given to the acupuncture group, while oral Yaotongning pills were given to the drug group. The entire effective rate of the acupuncture group is 91.23 percent, whereas the total effective rate of the pharmacological group is 80 percent, according to the findings. The pathogenesis of clinical lumbar intervertebral disc protrusion patients is mostly cold coagulation and blood stasis, and moxibustion has the effects of warming the meridians and dispelling cold, activating blood and dredging collaterals, so there are more reports of moxibustion. Literature [5] took Shenshu and Mingmen Fuzi cake moxibustion combined with massage to treat 17 patients with LIDP. Among them, 8 cases are cured, 5 cases are markedly effective, and 4 cases improved. The literature [6] randomly divided 74 patients with LIDP into a treatment group and a control group, with 37 cases in each group. The treatment group is treated with acupoint heat-sensitive suspension moxibustion, and the control group is treated with conventional acupuncture. The results showed that the total effective rate of the treatment group is 97.5%, and the total effective rate of the control group is 88.3%. The difference is statistically significant (*P* < 0.05). It shows that the clinical efficacy of thermal moxibustion in treating lumbar intervertebral disc protrusion is significantly better than that of conventional acupuncture.

The literature [7] used warm acupuncture to treat 50 cases of lumbar intervertebral disc protrusion. The results showed that 18 cases are cured, 22 cases are markedly effective, 8 cases are effective, and 2 cases are ineffective. The total effective rate is 96%. The conclusion shows that warm needling moxibustion has a good effect on lumbar intervertebral disc protrusion. The literature [8] treated 93 cases of lumbar intervertebral disc protrusion with warm needle all-in-one acupuncture, which was compared with 92 cases in the ordinary acupuncture group. The results showed that the total effective rates of the two groups are 95.70% and 82.61%, respectively. The warm-needle and combined acupuncture group had better efficacy than the ordinary acupuncture group. In the warm needling group, 74 cases are followed up, including 8 cases of recurrence. In the normal acupuncture group, 73 cases are followed up, of which 28 cases recurred. The half-year recurrence rates of the two groups are 10.81% and 38.36%, respectively, indicating that the warm needling and all-acupuncture group has a stable curative effect and a lower recurrence rate than the ordinary acupuncture group. The literature [9] used acupuncture plus moxa sticks to treat 80 patients with LIDP. As a result, 67 cases are cured, 9 cases improve, 4 cases are ineffective, and the total effective rate is 95%.

Numerous experimental research have revealed that acupuncture has a considerable impact in treating lumbar intervertebral disc protrusion. Acupuncture therapy for lumbar protrusion is thought to increase local blood circulation in the waist and legs, stimulate metabolism, and improve the interaction between the lumbar intervertebral disc protrusion and nerve roots, according to modern research. It also reduces nerve root inflammation and edema, loosens adhesions, and regulates peripheral and central nerve function as well as immunological activity and chemical inflammation-stimulating mediators [10]. The present clinical acupuncture therapy of lumbar protrusion is largely based on the local Huatuo Jiaji or Backshu acupoints, since the acupoints themselves have a therapeutic impact. Furthermore, in conjunction with the meridian treatment theory, patients who feel pain and numbness in the area where they follow the whole sun meridian should be provided with Chengfu, Weizhong, Chengshan, Kunlun, and other acupoints. Huantiao, Fengshi, Yanglingquan, Feiyang, Taichong, and other herbs may be utilized for patients with symptoms related to the foot-Shaoyang meridian. Patients with a variety of illnesses might benefit from combining the two meridians' major points.

In the literature [11], 97 cases of acute pain of lumbar disc herniation were treated by remote acupoint selection combined with ultrashort wave. The treatment group was treated with acupuncture of Weizhong, Yanglingquan Feiyang, and foot Ganoderma lucidum combined with ultrashort wave, while the control group was treated with acupuncture of Shenshu, qihaishu, Jiaji, Zhibian, Huantiao, and Weizhong. The results showed that the total effective rate of the treatment group was 96.08%, which was better than 78.26% of the control group. Acupuncture of Weizhong, Yanglingquan Feiyang, and foot Ganoderma lucidum was combined with ultrashort wave, while the control group was treated with acupuncture of Shenshu, qihaishu, Jiaji, Zhibian, Huantiao, and Weizhong. The results showed that the total effective rate of the treatment group was 96.08%, which was better than 78.26% of the control group. Acupuncture at the original points of the Sanyin meridian of the foot, Taichong, Taixi, Taibai, and the Sanyang meridian of the foot by using the method of matching the points of the original collaterals to acupuncture the protruding segments and upper and lower vertebrae Jiaji points, Shenshu, and Dachangshu on both sides are the main points, and the main points along the meridian of the affected limb are matched [12]. The results of the study show that the total effective rate of the treatment group is 96.7%, which is better than that of the control group 86.7%, and the VAS pain of the two groups of patients, both the score and the JOA score for low back pain, showed that the patient's symptoms improved significantly after treatment. In clinical practice, some doctors choose acupoints other than the fourteen meridians as the main acupoints for treatment, which can also achieve certain curative effects. In document [13], 70 patients with lumbar disc herniation were treated with acupuncture in the treatment group, Linggu, Dabai, Zhongbai, wrist Shun 1 and wrist Shun 2 points of Dongqi point, and acupuncture in the control group. For the clinically commonly used acupoints for lumbar protrusion, the results of the study showed that the total effective rate of the treatment group was 85.29%, which was higher than 70.59% of the control group. The acupuncture technique can also adjust the local benign stimulation of acupoints and even the body's body functions and has always been valued by clinical physicians. Literature [14] utilizes the dragon-tiger battle acupuncture technique, in which the doctor twists the thumb forward and left (clockwise) 9 times and then right and back (counterclockwise) 6 times after acupuncture acquires the air. The acupuncture approach was alternated with the traditional method of flattening, replenishing, and lowering acupuncture, and the results were compared. The study's findings revealed that the treatment group's overall effective rate was 93.3 percent, which was higher than the control group's 90 percent, and the difference was statistically significant. The traditional method of burning mountain fire to deeply puncture Jiaji points on the waist was used in the literature [15], and the results showed that when compared to the conventional method of flattening and relieving acupuncture, the total effective rates of the two groups were 97.5 percent and 82.5 percent, respectively. Literature [16] divided 54 patients into 3 groups randomly and then explored the curative effect of needle retention time for acupuncture treatment of lumbar protrusion. The results showed that the total effective rate of the 15-minute needle retention group was 68.75%, and the total effective rate of the 30-minute needle retention group was 88.89%, and the total effective rate of the 45-minute needle retention group was 94.44%. There was no significant difference in the pairwise comparison between the 3 groups, which provided a reference for improving the efficiency of clinical outpatient services.

## 3. Methods and Information

The symptoms and signs of the patient have the following characteristics. The patient has a clear history of chronic lumbar strain, trauma, or cold and damp invasion. The pain is mainly in the waist, or accompanied by pain and numbness in the buttocks, lower limbs, abdomen, and groin area, sacral tail, and perineum. Moreover, patients need to adopt forced postures such as scoliosis and slight knee flexion to relieve pain [4, 17]. The patient is accompanied by positive Lasegue sign, Lasegue enhancement sign, tenderness of the diseased vertebral body or paraspinous process, and even muscle atrophy. Patients may also have the corresponding obstacles to the motor and sensory functions of the innervating nerves, as well as the nerve reflexes, such as weakened dorsiflexion of the hallux, decreased sensation of the outer calf, and disappearance of the Achilles tendon reflex.

Modern medical imaging technology: X-ray shows scoliosis and narrowing of diseased intervertebral disc, or CT and MRI show intervertebral disc protrusion, protrusion and protrusion, which can be used as the basis of auxiliary diagnosis.

The study adopted a simple random method. The patients are assigned to the treatment group (acupuncture combined with massage group) and the control group (acupuncture only group) at a ratio of 1 : 1, 30 cases in each group, and then, the clinical efficacy is observed [18].

The treatment group was treated as follows:

Point selection is as follows: Ashi, Yaojiaji (double), Dachangshu (double), Shenshu (double), and Weizhong (double).

During the operation, the patient takes the prone position, disinfects the designated treatment site with 75% alcohol, and adopts the method of rapid needle insertion with one hand. Waist Jiaji points, Dachangshu points, and Shenshu points were directly pierced 0.8-1.2 inch. The Weizhong point was pierced 0.5-0.8 inch straight. After the needle is inserted, the needle needs to be kept for 30 minutes. The needles were retained for 30 minutes, and the needles were needled once every 10 minutes.

During the Tuina operation, after the patient was treated with rolling, pressing, spotting, and pressing methods to dredge the meridian points, followed by leg bending, waist pulling, and McKenzie therapy to correct the lesion and restore the original vertebral body function, (1) the patient took the prone position, and the therapist stands on the affected side [19]. The treatment started from the lower waist, along the bladder meridian, through the buttocks, the back of the thigh, to the back of the calf, back and forth 3 to 5 times. The patient was put on pillows on the chest and thighs to hang the abdomen, and the waist stretched back naturally. Acupoints such as Shenshu, Dachangshu, paraspinous tenderness point, Ju iliac, and Huantiao were pressed. The therapist overlapped his hands on the lower waist and performed 5 to 10 squeezing techniques. Then, the therapist tapped Chengfu, Yinmen, Weizhong, Chengshan, and other points and then ended the technique. (2) During the leg bending method, The patient lied on his back, and the therapist stranded on the side of the patient's limited leg. The therapist bent the patient's knees on his shoulders, asked the patient to push his thighs away from his shoulders for 6'10 seconds, and then relax. After the patient relaxes, he pushed the patient's thigh towards his shoulder to the end, maintaining a traction force for l0 seconds, but did not cause pain, and the operation was repeated 3 times [20, 21].

The therapist held the patient's shoulder with one hand to prepare for pushing back, while the other hand squeezed the elbow joint on the patient's buttocks to prepare for pushing forward, using the waist approach. The patient relaxed, and the therapist rotated the lumbar spine passively with both hands in various directions at the same time.

The control group was treated as follows:

(1) The acupoint selection is the same as the treatment group. (2) The operation, needle retention time, and replenishing and reducing techniques were the same as those in the treatment group. (4) Course of treatment: the above operations are performed once every other day, 3 times a week for diagnosis and treatment, 6 times as a course of treatment, a total of 2 courses of treatment. The curative effect will be evaluated after the course of treatment.

The visual analogue scale (VAS) approach was employed in the investigation. Each grid represents 1 point on a graph marked with a scale and evenly splits into l0 grids, with the two ends marked with “0” for “painless” and “10” for “severe pain.” In front of the patient, this image was presented. The patient was instructed to choose the scale that best represented their pain level at the moment, based on their personal pain assessment, and to accurately record the pain score.

The patient's pertinent research data and other data are gathered and entered into an Excel spreadsheet, and statistical analysis is performed using the SPSS 17.0 statistical program. The mean standard deviation will be used to describe the data related to the measurement data. The experiment uses a two independent samples *t* test on the data of two separate samples. The chi-square test may be used to examine data from the count data set. If it belongs to two groups of independent data, the Wilcoxon rank sum test comparison method is used in the experiment. If it is a strong paired data, the experiment uses the Wilcoxon signed rank test comparison method of the paired sample difference [22].

## 4. Result

The average course of disease in the treatment group is similar to that in the control group. Through the *t* test on the data of two independent samples, it is found that there was no difference in the mean course of the two groups of cases, as shown in Table 1.

The *t* test was used for the pain index scores of the two groups of patients before treatment. The results show that there was no difference in the VAS scores of the two groups before treatment, as shown in Table 2.

After treatment, the treatment group's effective rate was greater, and the total in the control group was lower than in the treatment group. On the curative impact comparison between the two groups of patients, the rank sum test was used. As shown in Table 3, the findings reveal that the H0 hypothesis is rejected, indicating that the overall effectiveness difference between the treatment and control groups is statistically significant.

The *t* test was used for the pain index scores of the two groups of patients before treatment. The results show that the VAS pain index scores of the two groups of cases are different after treatment, as shown in Table 4.

During the entire acupuncture treatment process, due to the advancement of acupuncture and moxibustion treatment related to the patient, the patient did not have any adverse reactions such as needle dizziness or stuck needles due to the first contact with acupuncture, or being in a nervous or hungry state. The safety evaluation of the treatment method is carried out on the two groups of patients, and the results obtained are shown in Table 5.

On the basis of the above research, the posttreatment satisfaction survey statistics of patients are obtained, and the results shown in Table 6 are obtained. From Table 6, it can be seen that the method proposed in this paper has higher satisfaction among the patient population.

## 5. Analysis and Discussion

Massage therapy is an important clinical treatment method of TCM. Under the guidance of TCM theory, doctors use specific techniques to directly stimulate the patients' meridian points or local Ashi points to achieve the purpose of treatment. Massage treatment, according to Chinese medicine, has the properties of dredging the meridians, reconciling qi and blood, and balancing yin and yang. It is one of the most common therapeutic options for lumbar intervertebral disc protrusion. Massage has been proven to have the functions of reducing nerve root compression, loosening adhesion, anti-inflammatory and analgesic, balance adjustment, strengthening human immunity, improving microcirculation and blood rheology, and restoring the balance of lumbar structure mechanics to achieve the goal of eliminating clinical symptoms and signs in modern studies. As a result, it is often employed in clinical practice. The mechanical equilibrium between the intervertebral discs is improved first. Massage therapy has been shown in studies to adjust the positional relationship between the intervertebral disc and the nerve root, and the adhered intervertebral disc tissue is loosened, promoting the recovery and reduction of the herniated intervertebral disc, effectively improving the symptoms of nerve root compression, and relaxing the tendons and dredging the collaterals. In addition, the lumbar spine's natural physiological curvature has been restored, and the distribution of force lines in the spine has been readjusted, restoring the spine's internal and exterior mechanical balance. It also has anti-inflammatory and analgesic properties. It may relax waist muscles, minimize systemic and local circulation disturbances, and relax local tenderness sites. This allows the local lymphatic vessels to widen, the local lymphatic circulation to improve, and the nutrition and metabolism of the local tissues to improve, all of which aid in the absorption and clearance of edema and inflammatory compounds in the local tissues. Third, it changes the shape of the protrusion and its relative positional relationship with the nerve root. In recent years, research has proved that the relative position of nerve roots has changed through massage therapy, so that the pressure and stimulation of the protruding nucleus pulposus on the nerve roots are relieved or even relieved. Moreover, the inflammatory adhesion between the protrusion and the nerve root is loosened, so as to achieve the purpose of changing the relative position between the intervertebral disc and the nerve root. Fourth, it relieves the symptoms of secondary compression. The lumbar and leg pain caused by lumbar intervertebral disc protrusion can be considered as primary entrapment is the compression of the nerve root by the protrusion. Under the action of external force, the compression of the lower nerve is called secondary entrapment. Only when the primary compression and secondary compression have a certain degree of influence on the nerves will clinical symptoms appear. Therefore, we can use massage techniques to treat lumbar intervertebral disc herniation from the removal of primary entrapment. At the same time, we can focus on loosening the points where nerve roots are prone to compression to gradually relieve the patient's symptoms and signs, and even disappear, so as to achieve the purpose of time-saving and efficient treatment.

Pain and dysfunction of the waist and legs are the most common clinical signs of lumbar intervertebral disc herniation. The therapy is founded on the notion of not exacerbating pain and adopting pain-relieving postures and activities. Manual reduction, unlike traditional reduction techniques in the past, can cause the intervertebral space, the annulus fibrosus, and the posterior longitudinal ligament to rotate and traction in response to the protruding nucleus pulposus, causing peripheral pressure to be generated and the protrusion to be accommodated. But manual reduction often aggravates pain and symptoms, and it is not unusual for new injuries to occur as a result. McKenzie treatment is preferable because of its foundation in spinal biomechanics. The procedure is especially useful when the etiology of lumbar intervertebral disc protrusion patients is caused by the contact between the inside and outside of the spinal canal. It may relax the muscles that have been stressed by spasms and restore the nucleus pulposus's proper displacement, resulting in pain relief.

For patients with lumbar intervertebral disc protrusion, acupuncture can improve the blood circulation of the diseased area and accelerate the metabolism between tissue cells and anti-inflammatory and analgesic. When it is combined with massage techniques, it has the effect of reducing nerve root compression and loosening adhesion. When it is recombined with McKenzie therapy, the muscles that are strained by spasm are relaxed, and the prominent nucleus pulposus is restored.

## 6. Conclusion

Lumbar intervertebral disc herniation is a frequently occurring disease in modern social life. It has a serious impact on the quality of daily life and psychosocial burden of patients and has attracted the attention of the public. This topic summarizes the current status of traditional Chinese medicine and Western medicine treatment of lumbar intervertebral disc protrusion and combs the related literature research on acupuncture, McKenzie therapy, and massage. This time, acupuncture combined with McKenzie and massage therapy was used to treat lumbar intervertebral disc protrusion. Compared with the control group using the conventional acupuncture method, it provides a more effective treatment plan for improving the clinical diagnosis and treatment of lumbar intervertebral disc protrusion.

## Figures and Tables

**Table 1:** Comparison of disease course before treatment.

Number	Control group	Test group	Number	Control group	Test group
1	19.83	18.25	17	19.76	19.25
2	18.72	19.68	18	18.29	18.89
3	18.88	19.02	19	19.57	19.32
4	18.68	18.42	20	19.95	18.82
5	18.18	18.35	21	19.75	19.76
6	19.62	19.46	22	19.40	18.72
7	19.00	18.08	23	19.47	19.14
8	19.02	19.33	24	19.00	18.95
9	19.80	19.83	25	19.57	18.42
10	19.33	18.90	26	18.10	19.48
11	18.84	18.02	27	19.42	18.25
12	19.07	19.05	28	19.24	19.77
13	18.26	18.63	29	18.04	19.94
14	19.43	19.01	30	18.71	19.91
15	18.83	18.84	31	18.65	19.41
16	18.33	19.55	32	19.93	18.93

**Table 2:** VAS score before treatment.

Number	Control group	Test group	Number	Control group	Test group
1	4.52	5.30	17	6.10	6.42
2	4.46	6.35	18	4.67	4.88
3	6.23	4.58	19	3.65	4.62
4	4.82	6.09	20	5.12	5.07
5	6.78	4.69	21	5.44	5.11
6	3.87	4.96	22	4.01	5.23
7	6.76	4.97	23	6.08	6.50
8	5.40	5.28	24	5.19	5.31
9	7.16	4.90	25	7.00	4.92
10	3.86	6.07	26	3.65	4.76
11	3.90	6.48	27	5.97	4.73
12	7.04	6.20	28	6.36	6.60
13	4.96	6.48	29	5.01	6.45
14	5.84	6.35	30	6.03	4.61
15	6.29	5.13	31	3.87	5.23
16	3.98	5.42	32	7.04	4.49

**Table 3:** Comparison of the overall efficacy of the two groups of patients.

Number	Control group	Test group	Number	Control group	Test group
1	84.46	96.14	17	83.36	95.83
2	84.90	95.40	18	84.20	96.27
3	83.13	96.68	19	83.69	95.26
4	84.45	95.51	20	83.99	97.37
5	84.78	97.44	21	84.52	95.03
6	83.60	96.88	22	83.64	95.60
7	83.82	96.22	23	83.89	97.65
8	83.90	96.36	24	84.18	96.44
9	83.70	96.47	25	83.23	96.26
10	84.21	97.54	26	83.01	95.54
11	84.03	97.85	27	84.31	97.36
12	84.94	95.84	28	83.11	95.66
13	83.43	96.74	29	84.79	97.60
14	83.95	95.16	30	83.05	97.24
15	84.72	96.88	31	83.52	97.80
16	84.94	97.93	32	84.24	96.23

**Table 4:** Comparison of VAS scores between the two groups of patients after treatment.

Number	Control group	Test group	Number	Control group	Test group
1	1.29	0.80	17	2.57	0.61
2	3.86	0.84	18	1.24	2.67
3	1.03	2.39	19	1.23	1.18
4	3.14	0.62	20	2.65	1.69
5	3.44	1.58	21	2.97	0.37
6	1.89	1.65	22	1.73	1.43
7	3.38	1.45	23	1.40	2.98
8	3.28	2.92	24	3.35	2.48
9	2.56	0.31	25	4.00	0.22
10	2.70	0.27	26	3.96	2.18
11	1.74	0.38	27	2.95	2.92
12	2.52	1.48	28	2.03	1.46
13	2.82	1.11	29	1.40	2.99
14	3.76	0.84	30	1.62	1.13
15	3.30	2.12	31	2.66	1.60
16	1.54	1.28	32	3.77	1.09

**Table 5:** Safety evaluation of treatment methods.

Number	Control group	Test group	Number	Control group	Test group
1	73.68	89.53	17	75.83	92.18
2	77.18	93.56	18	76.61	92.60
3	74.39	90.92	19	74.29	92.45
4	78.22	93.41	20	72.32	89.48
5	72.76	93.63	21	73.26	91.44
6	72.45	92.96	22	76.46	91.00
7	75.22	93.63	23	72.67	91.66
8	76.04	93.54	24	73.69	91.01
9	77.71	92.83	25	76.00	90.81
10	78.58	89.86	26	76.05	93.47
11	71.57	93.32	27	71.16	91.21
12	72.33	92.73	28	78.51	91.80
13	77.25	89.63	29	77.59	89.35
14	73.92	93.34	30	74.70	92.54
15	72.75	92.00	31	76.50	92.07
16	74.49	92.03	32	74.34	93.81

**Table 6:** Patient satisfaction survey.

Number	Control group	Test group	Number	Control group	Test group
1	84.48	95.10	17	85.72	96.84
2	87.37	95.11	18	82.57	94.65
3	89.15	96.97	19	85.86	96.02
4	84.66	96.53	20	87.10	96.42
5	83.09	95.35	21	87.97	95.16
6	81.69	94.24	22	82.77	95.66
7	80.87	96.07	23	89.03	94.96
8	85.85	95.50	24	80.19	95.36
9	80.17	96.94	25	89.76	95.51
10	82.08	97.47	26	89.49	97.23
11	87.26	96.18	27	82.98	95.87
12	85.92	97.23	28	88.64	97.40
13	87.95	93.30	29	89.42	97.15
14	90.46	95.47	30	79.47	97.20
15	85.75	97.57	31	85.39	97.60
16	79.96	94.69	32	79.50	94.65

## Data Availability

The data used to support the findings of this study are included within the article.

## References

[1] Ning H. X., Yuan Y. W., Zhang Q. Y., Sun Z. Z., Ning H. Y., Wang P. (2018). Percutaneous transforaminal endoscopic discectomy and miniincision surgery in the treatment of lumbar intervertebral disc protrusion. *Journal of Biological Regulators and Homeostatic Agents*.

[2] Wu G. N., Zhang S. M., Jin J., Sun B. Q. (2017). Percataneous endoscopic lumbar discectomy for the treatment of lumbar intervertebral disc protrusion. *Zhongguo gu shang= China journal of orthopaedics and traumatology*.

[3] Song H. P., Sheng H. F., Xu W. X. (2017). A case-control study on the treatment of protrusion of lumbar intervertebral disc through PELD and MED. *Experimental and Therapeutic Medicine*.

[4] Zhang B., Xu H., Wang J., Liu B., Sun G. (2017). A narrative review of non-operative treatment, especially traditional Chinese medicine therapy, for lumbar intervertebral disc herniation. *Bioscience Trends*.

[5] Zhang B., Guo W., Sun C. (2018). Dysregulated MiR-3150a-3p promotes lumbar intervertebral disc degeneration by targeting aggrecan. *Cellular Physiology and Biochemistry*.

[6] Tao X. Z., Jing L., Li J. H. (2018). Therapeutic effect of transforaminal endoscopic spine system in the treatment of prolapse of lumbar intervertebral disc. *European Review for Medical and Pharmacological Sciences*.

[7] Asiri F., Tedla J., Alshahrani M. D., Ahmed I., Reddy R., Gular K. (2020). Effects of patient-specific three-dimensional lumbar traction on pain and functional disability in patients with lumbar intervertebral disc prolapse. *Nigerian Journal of Clinical Practice*.

[8] Rade M., Pesonen J., Könönen M. (2017). Reduced spinal cord movement with the straight leg raise test in patients with lumbar intervertebral disc herniation. *Spine*.

[9] Tang S., Mo Z., Zhang R. (2018). Acupuncture for lumbar disc herniation: a systematic review and meta-analysis. *Acupuncture in Medicine*.

[10] Mahatthanatrakul A., Kotheeranurak V., Lin G. X., Hur J. W., Chung H. J., Kim J. S. (2019). Comparative analysis of the intervertebral disc signal and annulus changes between immediate and 1-year postoperative MRI after transforaminal endoscopic lumbar discectomy and annuloplasty. *Neuroradiology*.

[11] Gwak G. T., Hwang U. J., Jung S. H., Kim H. A., Kim J. H., Kwon O. Y. (2019). Comparison of MRI cross-sectional area and functions of core muscles among asymptomatic individuals with and without lumbar intervertebral disc degeneration. *BMC Musculoskeletal Disorders*.

[12] Ohnishi T., Sudo H., Tsujimoto T., Iwasaki N. (2018). Age-related spontaneous lumbar intervertebral disc degeneration in a mouse model. *Journal of Orthopaedic Research®*.

[13] Duran S., Cavusoglu M., Hatipoglu H. G., Cılız D. S., Sakman B. (2017). Association between measures of vertebral endplate morphology and lumbar intervertebral disc degeneration. *Canadian Association of Radiologists Journal*.

[14] Tang G., Wang Z., Chen J., Zhang Z., Qian H., Chen Y. (2018). Latent infection of low-virulence anaerobic bacteria in degenerated lumbar intervertebral discs. *BMC Musculoskeletal Disorders*.

[15] Singh S., Kumar S., Chahal G., Verma R. (2017). Selective nerve root blocks vs. caudal epidural injection for single level prolapsed lumbar intervertebral disc - A prospective randomized study. *Journal of clinical orthopaedics and trauma*.

[16] Yang L., Lu H. H. (2017). Value of a new pathological classification of lumbar intervertebral disc herniation based on transforaminal endoscopic observations. *Experimental and Therapeutic Medicine*.

[17] Lurie J. D., Henderson E. R., McDonough C. M. (2016). The effect of expectations on treatment outcome for lumbar intervertebral disc herniation. *Spine*.

[18] Millecamps M., Stone L. S. (2018). Delayed onset of persistent discogenic axial and radiating pain after a single-level lumbar intervertebral disc injury in mice. *Pain*.

[19] Feng X., Jiang Q., Zhang Y. (2022). Pediatric Tuina in children with autism spectrum disorder: a study protocol for a randomized controlled trial. *Trials*.

[20] Farrokhi M. R., Karimi M. H., Ghaffarpasand F., Sherafatian M. (2020). MicroRNA-199a Upregulation mediates lumbar intervertebral disc degeneration and is associated with clinical grades of degeneration. *Turkish Neurosurgery*.

[21] Chen J., Liu T. Y. (2019). Quantitative research technology of tuina manipulations. *Journal of Acupuncture and Tuina Science*.

[22] Hu Y., Tang J. S., Hou S. X. (2017). Neuroprotective effects of curcumin alleviate lumbar intervertebral disc degeneration through regulating the expression of iNOS, COX-2, TGF-*β*1/2, MMP-9 and BDNF in a rat model. *Molecular Medicine Reports*.

